# Effects of Different Doses of Dexmedetomidine Combined with Thoracic Paravertebral Nerve Block Anesthesia on Agitation and Hemodynamics in Patients Undergoing Thoracotomy during Recovery

This article has been retracted.

**DOI:** 10.1155/2022/7804584

**Published:** 2022-06-29

**Authors:** Baoli Zu, Yong Yang, Shengchi Shi

**Affiliations:** ^1^Department of Anesthesiology, Guizhou International General Hospital, Guiyang, China; ^2^Department of Anesthesiology, First Affiliated Hospital of Army Military Medical University, Chongqing, China

## Abstract

**Objective:**

To investigate the effect of different doses of dexmedetomidine combined with thoracic paravertebral nerve block anesthesia on agitation and hemodynamics in patients undergoing thoracotomy during recovery.

**Methods:**

One hundred patients who underwent thoracotomy in our hospital from August 2018 to April 2021 were enrolled and assigned (1 : 1 : 1 : 1) into 4 groups via the random number table method. The patients in the control group were treated with double-lumen tube general anesthesia + ropivacaine for thoracic paravertebral nerve block anesthesia; patients in experimental group A received double-lumen general anesthesia +0.5 *μ*g·kg^−1^ dexmedetomidine + ropivacaine for thoracic paravertebral nerve block anesthesia; patients in experimental group B received thoracic paravertebral nerve block anesthesia with double-lumen general anesthesia +1.0 *μ*g·kg^−1^ dexmedetomidine + ropivacaine; patients in experimental group C received thoracic paravertebral nerve block anesthesia with double-lumen general anesthesia +1.5 *μ*g·kg^−1^ dexmedetomidine + ropivacaine. The postoperative recovery time and visual analog scale (VAS), level of hemodynamics (heart rate (HR), mean arterial pressure (MAP)), agitation during the recovery period, and complications were compared amongst the 4 groups of patients at different time points.

**Results:**

The postoperative VAS scores of patients in groups B2 and B3 were slightly lower than those of patients in groups A and B1, but a one-way analysis of variance revealed no statistical difference in the postoperative recovery time and VAS pain scores of the four groups (*P* > 0.05), and the recovery time of patients in experimental group C was slightly higher than that of patients in group B2. At T0 and T1, there was no significant difference in the levels of HR and MAP among the four groups (*P* > 0.05). The levels of HR and MAP of the patients in groups B2 and B3 were significantly different from the patients in the control group and experimental group A at T2 and T3 (*P* < 0.05). The patients in experimental group B and experimental group C showed better outcomes than those in the control group and experimental group A in the assessment of agitation during the recovery period (*P* < 0.05). There was no significant difference in the incidence of complications among the four groups (*P* > 0.05).

**Conclusion:**

In line with the principle of preference for a small anesthesia dose, 1.0 *μ*g·kg^−1^ dose of dexmedetomidine combined with ropivacaine produces a pronounced efficacy in patients undergoing thoracotomy. It effectively controls the occurrence of agitation during the recovery period and maintains the stability of the patient's hemodynamics, with a high clinical safety profile.

## 1. Introduction

Thoracotomy is one of the common surgical methods in clinical practice, and it is applied in the following conditions: (1) active bleeding in the thoracic cavity and a drop in blood pressure; (2) tension pneumothorax and bronchial rupture; the drainage bottle continues to overflow a lot, and the lung still does not expand; (3) coughing up blood continuously; (4) those with heart and large blood vessel damage; (5) rupture of the diaphragm and rupture of the esophagus; (6) closed repair of large open chest wall injuries; (7) early clearance of hemothorax, there are a large number of hemothorax, but the drainage is not smooth, and there is suspected intrathoracic blood clot; (8) poor antishock effect. Pulmonary complications often occur in patients undergoing thoracotomy due to the characteristics of the surgical site, method, and underlying disease. It is associated with body circulatory dysfunction during recovery from anesthesia and cardiovascular and other adverse events due to the surgery-related trauma and endotracheal intubation [1, 2]. Thoracic paravertebral nerve block anesthesia is a commonly used anesthesia method in thoracic surgery, with a high safety profile. It is also conducive to maintaining hemodynamic stability and analgesic effect [3]. Ropivacaine is a commonly used local anesthesia drug characterized by convenient use and ideal analgesic effect, while dexmedetomidine is a highly selective adrenergic *α*_2_ receptor agonist with a good efficacy profile in antianxiety, sedation, and analgesia [4]. It is acknowledged that with the combination with long-acting amide local anesthetics, the analgesic effect can be further enhanced [5]. Patients are vulnerable to complications such as choking, agitation, tachycardia, and elevated blood pressure when removing the tracheal tube and in the course of the recovery period during thoracic surgery [6]. There is an urgent need to develop effective therapeutic strategies to counteract these rising trends. Accordingly, the principal objective of the present study was to investigate the impact of different doses of dexmedetomidine combined with thoracic paravertebral nerve block anesthesia on agitation and hemodynamics in patients undergoing thoracotomy during recovery.

## 2. Materials and Methods

### 2.1. Baseline Data

One hundred patients who underwent thoracotomy in our hospital from August 2018 to April 2021 were enrolled and assigned (1 : 1 : 1 : 1) into 4 groups via the random number table method. The patients in the control group were treated with double-lumen tube general anesthesia + ropivacaine for thoracic paravertebral nerve block anesthesia; patients in experimental group A received double-lumen general anesthesia +0.5 *μ*g·kg^−1^ dexmedetomidine + ropivacaine for thoracic paravertebral nerve block anesthesia; patients in experimental group B received thoracic paravertebral nerve block anesthesia with double-lumen general anesthesia +1.0 *μ*g·kg^−1^ dexmedetomidine + ropivacaine; patients in experimental group C received thoracic paravertebral nerve block anesthesia with double-lumen general anesthesia +1.5 *μ*g·kg^−1^ dexmedetomidine + ropivacaine. There were 18 males and 7 females in the control group, aged 48–66 years, with an average age of (56.62 ± 5.21) years. There were 17 males and 8 females in group B1; the age ranged from 47 to 66 years, with an average age of (56.57 ± 5.30) years. There were 19 males and 6 females in group B2, aged 47–65 years, with an average age of (56.48 ± 5.17) years. There were 16 males and 9 females in group B3; the age ranged from 49 to 68 years, with an average age of (56.70 ± 5.30) years. Patients with diabetes, metabolic disorders, and obstructive pulmonary diseases were excluded from the study. The study was conducted in strict accordance with the protocol of the Clinical Trial Ethics Committee of our hospital, and all patients and their families consented to participate in this study.

### 2.2. Methods

After entering the operating room, all patients underwent routine electrocardiogram, transradial cannulation was performed under local anesthesia, and central venous access was established. The patient was assisted to perform lateral recumbency and routinely sterilized, and ultrasound-guided thoracic paravertebral nerve block was performed on the affected side using a sterile protective cover to protect the ultrasound probe [7]. After local anesthesia with 1% lidocaine at a point 2.5 cm away from the T6 spinous process, a single-point block was selected, and the needle was held in the right hand to perform thoracic paravertebral long-axis in-plane technical puncture to confirm that the needle tip reached the paravertebral space to inject local anesthesia [8]. The control group was injected with 20 mL of 0.5% ropivacaine alone; experimental group A was injected with 0.5 *μ*g·kg^−1^ dexmedetomidine combined with ropivacaine; experimental group B was injected with 1.0 *μ*g·kg^−1^ dexmedetomidine combined with ropivacaine; experimental group C was injected with 1.5 *μ*g·kg^−1^ dexmedetomidine combined with ropivacaine. After the nerve block was completed, the alcohol cotton ball test was used to detect the temperature and touch of the skin in the corresponding area and then determine whether the nerve block was successful [9].

Anesthesia induction was started 10 min after confirmation of a successful block. Induction of anesthesia: 0.06–0.14 mg·kg^−1^ midazolam (Jiangsu Nhwa Pharmaceutical Co., Ltd., H20031037), 0.4–0.6 *μ*g·kg^−1^ sufentanil (Yichang Renfuyao Industry Co., Ltd., H20054172), 1.8–2.6 mg·kg^−1^ propofol (AstraZeneca Co., Ltd., H20083107), and 0.10 mg·kg^−1^ cis-atracurium (Xianju Pharmaceutical Co., Ltd., H20060869) were injected for intravenous induction. A double-lumen bronchial catheter was then inserted orally, positioned with a fiberoptic bronchoscope, and the patient was mechanically ventilated after tracheal intubation. Anesthesia maintenance: 2–6 mg/(kg·h) propofol (Sichuan Guorui Pharmaceutical Co., Ltd., H20040079) and 0.10–0.20 *μ*g/(kg·min) remifentanil (Yichang Renfu Pharmaceutical Co., Ltd., H20143314) were given via intravenous infusion, and cis-Atracurium was intermittently injected to maintain the heart rate (HR) and mean arterial pressure (MAP) fluctuations that do not exceed 25% of the baseline value. The intravenous analgesia pump was connected when the patient left the resuscitation room 1 h after the operation [10].

### 2.3. Observation Indicators

Vital signs (body temperature, respiration, pulse, blood pressure) at 10 minutes after the patient entered the room (T0), before anesthesia induction (T1), after tracheal intubation (T2), during skin incision (T3), and during extubation (T4) were monitored [11]. (1) Wake-up time was recorded by the medical staff of our hospital. (2) The visual analog scale (VAS) was used to evaluate the pain, with a total score of 10 points. The higher the patient's score, the more severe the pain. (3) Level of hemodynamics (heart rate (HR), mean arterial pressure (MAP)) was observed by the medical staff in our hospital. (4) Agitation during recovery was categorized as follows: Grade 0: the patient is calm and cooperative, is easy to wake up, and can follow verbal commands; Grade I: the patient is mildly restless, but can follow verbal commands; Grade II: the patient is very agitated, and verbal dissuasion is ineffective to make them calm down, are corresponding measures are needed; Grade III: the patient is restless, with intentions such as extubation and attacking medical staff. (5) Complications include nausea and vomiting, bradycardia, and hypotension [12].

### 2.4. Statistical Methods

All data analyses were performed with SPSS21.0 software. Measurement data are expressed as (*x* ± *s*), and the differences were analyzed using one-way analysis of variance followed by independent samples *t*-test; enumeration data are expressed as number of cases (rate), and the chi-square test was used for comparison. All tests were 2-sided, with a significance level of 0.05.

## 3. Results

### 3.1. Baseline Information

The baseline data of the four groups of patients were comparable (*P* > 0.05) (Table 1).

### 3.2. Recovery Time and VAS Pain Score

The postoperative VAS scores of patients in groups B2 and B3 were slightly lower than those of patients in groups A and B1, but one-way analysis of variance revealed no statistical difference in the postoperative recovery time and VAS pain scores of the four groups (*P* > 0.05), and the recovery time of patients in experimental group C was slightly higher than that of patients in experimental group B (Table 2).

### 3.3. Hemodynamics Levels at Different Time Points

At T0 and T1, there was no significant difference in the levels of HR and MAP among the four groups (*P* > 0.05). The levels of HR and MAP of the patients in groups B2 and B3 were significantly different from the patients in the control group and experimental group A at T2 and T3 (*P* < 0.05), as shown in Table 3.

### 3.4. Agitation Assessments during Recovery

The patients in experimental group B and experimental group C showed better outcomes than those in the control group and experimental group A in the assessment of agitation during the recovery period (*P* < 0.05), as shown in Table 4.

### 3.5. Complications

There was no significant difference in the incidence of complications among the four groups (*P* > 0.05), as shown in Table 5.

## 4. Discussion

Recent years witness an increasingly rising incidence of lung diseases in China, and multiple risk factors have been identified as contributors to the lung diseases; accordingly, the list is highly heterogeneous such as smoking, environmental pollution, and family history [13]. Surgery is the mainstay for its patients, and intraoperative thoracic paravertebral nerve block combined with general anesthesia is widely used in clinical thoracic surgery. The method has a good auxiliary analgesic effect and high drug safety, yet the patient is prone to adverse reactions or complications of anesthesia during operation and after the operation due to the rapid changes in hemodynamics during the recovery period [14]. Therefore, it is of utmost significance to reduce extubation-related cardiovascular stress response in patients undergoing thoracic paravertebral nerve block anesthesia to ensure the stable recovery of patients, which has profound implications for the prognosis of patients [15].

Ropivacaine is one of the commonly used long-acting amide local anesthetics, and it mainly acts by blocking the flow of sodium ions into the nerve fiber cell membrane [16], thereby producing a reversible blocking effect on the impulse conduction along with the nerve fiber. To our understanding, dexmedetomidine has a pronounced role in reducing the reactivity of patients, preventing bronchospasm, and reducing the occurrence of symptoms such as coughing during recovery, which can ensure the smooth progress of extubation during recovery. However, the clinical dose of dexmedetomidine remains controversial [17].

In line with our hypotheses, we found that the postoperative VAS scores of patients in groups B2 and B3 were slightly lower than those of patients in groups A and B1, but one-way analysis of variance revealed no statistical difference in the postoperative recovery time and VAS pain scores of the four groups and the recovery time of patients in experimental group C was slightly higher than that of patients in group B. Similarly, at T0 and T1, there was no significant difference in the levels of HR and MAP among the four groups. The levels of HR and MAP of the patients in groups B and C were significantly different from the patients in the control group and experimental group A at T2 and T3. Also in keeping with our hypotheses, the patients in experimental group B and experimental group C showed better outcomes than those in the control group and experimental group A in the assessment of agitation during the recovery period. Interestingly, there was no significant difference in the incidence of complications among the four groups. These findings suggest that ropivacaine alone and 0.5 *μ*g·kg^−1^ dexmedetomidine plus ropivacaine cannot effectively inhibit the intubation reaction of patients during surgery, while the doses of 1.0 *μ*g·kg^−1^ and 1.5 *μ*g·kg^−1^ dexmedetomidine plus ropivacaine can effectively reduce and control hemodynamics [18]. This may have been due to that the doses of 1.0 *μ*g·kg^−1^ and 1.5 *μ*g·kg^−1^ dexmedetomidine play a key role in reducing and controlling the stress response of patients. In addition, the postoperative VAS score, postoperative recovery time, and incidence of adverse reactions in experimental groups B and C were not significantly different from those in the control group and experimental group B. This would suggest that 1.0 *μ*g·kg^−1^ and 1.5 *μ*g·kg^−1^ doses of dexmedetomidine combined with ropivacaine exert good sedative and analgesic effects, without prolonging the recovery time of patients or raising the risk of complications [19]. The possible mechanism is that (1) dexmedetomidine, as a *μ*-opioid receptor agonist, can effectively block the release of norepinephrine, thereby weakening nerve signal transmission and ultimately reducing postoperative adverse symptoms such as hyperalgesia [18]; (2) dexmedetomidine can also reduce interleukin and inflammatory factors such as tumor necrosis factors, reduce the excitability of nerves, and thus reduce the pain of patients [19]; (3) dexmedetomidine can enhance the sympathetic nerve activity of patients and inhibit the occurrence of postoperative hyperalgesia from both positive and negative aspects [20]; (4) dexmedetomidine also has a certain antinociceptive effect, which further relieves pain and improves the sedation degree of patients [21].

To sum up, in line with the principle of preference of small anesthesia dose, a 1.0 *μ*g·kg^−1^ dose of dexmedetomidine combined with ropivacaine produces a pronounced efficacy in patients undergoing thoracotomy. It effectively controls the occurrence of agitation during the recovery period and maintains the stability of the patient's hemodynamics, with a high clinical safety profile.

## Figures and Tables

**Table 1:** Baseline data (n (%)).

	Control group (*n* = 25)	Experimental group A (*n* = 25)	Experimental group B (*n* = 25)	Experimental group C (*n* = 25)
Gender		^*∗*^	^*∗*^	^*∗*^
Male	18	17	19	16
Female	7	8	6	9
Age (year)	$\bar{x}\pm s$	$\bar{x}\pm s$	$\bar{x}\pm s$	$\bar{x}\pm s$
Mean age (year)	56.62 ± 5.21	56.57 ± 5.30	56.48 ± 5.17	56.70 ± 5.30

*Note.* ^*∗*^The gender and average age of the group were compared with those of the control group, and the difference was not statistically significant, *P* > 0.05.

**Table 2:** Comparison of wake-up time and VAS pain score ($\bar{x}\pm s$).

Groups	Postoperative recovery time (min)	VAS (point)
Control group (*n* = 25)	11.53 ± 4.62	2.53 ± 1.11
Experimental group A (*n* = 25)	13.02 ± 3.23	2.33 ± 1.04
Experimental group B (*n* = 25)	12.75 ± 3.68	2.05 ± 0.72
Experimental group C (*n* = 25)	14.11 ± 4.02	1.94 ± 0.67
*F*	1.827	2.187
*P*	0.147	0.095

**Table 3:** Comparison of hemodynamic (heart rate (HR), mean arterial pressure (MAP)) levels in different time periods ($\bar{x}\pm s$).

	Groups	T0	T1	T2	T3	T4
HR	Control group (*n* = 25)	85.11 ± 9.30	84.12 ± 11.01	86.50 ± 10.11	69.41 ± 8.02^*∗*^	60.53 ± 8.32^*∗*^
	Experimental group A (*n* = 25)	84.62 ± 9.71	81.70 ± 11.52	85.92 ± 10.31	65.10 ± 7.33^*∗*^	61.21 ± 7.92^*∗*^
	Experimental group B (*n* = 25)	84.20 ± 10.02	79.52 ± 10.80	70.22 ± 8.33^#@^	62.42 ± 7.04^*∗*^^#^	58.03 ± 7.53^*∗*^^#^
	Experimental group C (*n* = 25)	83.72 ± 9.12	78.81 ± 11.42	68.41 ± 8.13^#@^	53.51 ± 8.71^*∗*^^#@^	52.12 ± 8.43^*∗*^^#@^

MAP	Control group (*n* = 25)	90.21 ± 10.32	89.53 ± 12.31	94.12 ± 12.02	70.22 ± 7.52^*∗*^	68.72 ± 10.21^*∗*^
	Experimental group A (*n* = 25)	89.50 ± 11.03	87.92 ± 12.03	92.10 ± 12.73	72.63 ± 8.13^*∗*^	69.71 ± 10.63^*∗*^
	Experimental group B (*n* = 25)	90.71 ± 10.80	88.73 ± 11.94	78.51 ± 10.33^#@^	66.31 ± 6.52^*∗*^^#^	70.51 ± 9.62^*∗*^^#^
	Experimental group C (*n* = 25)	89.72 ± 10.51	86.42 ± 10.51	77.10 ± 10.52^#@^	62.43 ± 8.32^*∗*^^#@^	64.11 ± 9.82^*∗*^^#@^

*Note.* ^#^Comparison with T0 and T1, *P* < 0.05; ^*∗*^comparison with T2, *P* < 0.05; ^@^comparison with a control group and group B1, *P* < 0.05.

**Table 4:** Comparison of agitation during recovery (n (%)).

Groups	Grade 0	Grade I	Grade II	Grade III	Total incidence (%)
Control group (*n* = 25)	18	4	2	1	7 (28%)
Experimental group A (*n* = 25)	19	5	1	0	6 (24%)
Experimental group B (*n* = 25)	24	1	0	0	1 (4%)
Experimental group C (*n* = 25)	24	1	0	0	1 (4%)

**Table 5:** Comparison of complications (n(%)).

Groups	Nausea and vomiting	Bradycardia	Low blood pressure	Incidence (%)
Control group (*n* = 25)	2	1	2	5 (20%)
Group B1 (*n* = 25)	2	0	1	3 (12%)
Group B2 (*n* = 25)	1	1	0	2 (8%)
Group B3 (*n* = 25)	0	2	0	2 (8%)

## Data Availability

No data were used to support this study.
